RETRACTED

# Carbon monoxide inhibits Fas activating antibody-induced apoptosis in endothelial cells

**DOI:** 10.1186/2045-9912-1-8

**Published:** 2011-05-18

**Authors:** Xue Wang, Yong Wang, Seon-Jin Lee, Hong Pyo Kim, Augustine MK Choi, Stefan W Ryter

**Affiliations:** 1 Pulmonary, Allergy, and Critical Care Medicine, Department of Medicine, University of Pittsburgh Medical Center, Pittsburgh, PA 15213, USA; 2 Pulmonary and Critical Care Medicine, Brigham and Women's Hospital, Harvard Medical School, 75 Francis Street, Boston, MA, 02115, USA; 3 School of Biological Sciences, College of Natural Sciences, University of Ulsan, Ulsan, 680-749, Korea

## Abstract

**Background:**

The extrinsic apoptotic pathway initiates when a death ligand, such as the Fas ligand, interacts with its cell surface receptor (*ie*., Fas/CD95), forming a death-inducing signaling complex (DISC). The Fas-dependent apoptotic pathway has been implicated in several models of lung or vascular injury. Carbon monoxide, an enzymatic product of heme oxygenase-1, exerts antiapoptotic effects at low concentration *in vitro *and *in vivo*.

**Methods:**

Using mouse lung endothelial cells (MLEC), we examined the antiapoptotic potential of carbon monoxide against apoptosis induced by the Fas/CD95-activating antibody (Jo2). Carbon monoxide was applied to cell cultures *in vitro*. The expression and/or activation of apoptosis-related proteins and signaling intermediates were determined using Western Immunoblot and co-immunoprecipitation assays. Cell death was monitored by lactate dehydrogenase (LDH) release assays. Statistical significance was determined by student T-test and a value of *P *< 0.05 was considered significant.

**Results:**

Treatment of MLEC with Fas-activating antibody (Jo2) induced cell death associated with the formation of the DISC, and activation of caspases (-8, -9, and -3), as well as the pro-apoptotic Bcl-2 family protein Bax. Exposure of MLEC to carbon monoxide inhibited Jo2-induced cell death, which correlated with the inhibition of DISC formation, cleavage of caspases-8, -9, and -3, and Bax activation. Carbon monoxide inhibited the phosphorylation of the Fas-associated death domain-containing protein, as well as its association with the DISC. Furthermore, carbon monoxide induced the expression of the antiapoptotic protein FLIP and increased its association with the DISC.

CO-dependent cytoprotection against Fas mediated apoptosis in MLEC depended in part on activation of ERK1/2-dependent signaling.

**Conclusions:**

Carbon monoxide has been proposed as a potential therapy for lung and other diseases based in part on its antiapoptotic effects in endothelial cells. In vitro, carbon monoxide may inhibit both Fas/caspase-8 and Bax-dependent apoptotic signaling pathways induced by Fas-activating antibody in endothelial cells. Strategies to block Fas-dependent apoptotic pathways may be useful in development of therapies for lung or vascular disorders.

RETRACTED

## Background

Apoptosis, a form of programmed cell death, serves a critical function in the maintenance of tissue homeostasis under physiological conditions, as a component of developmental programs. Dysregulation of apoptosis may contribute to the progression of a number of disease states, including cancer, autoimmunity, and neurodegenerative disorders [1,2]. Furthermore, apoptosis has also been implicated in the pathogenesis of several pulmonary diseases, including acute lung injury/acute respiratory distress syndrome (ALI/ARDS) [3,4], and chronic obstructive pulmonary disease [5].

Apoptosis requires the regulated activation of proteases (*ie*., caspases) and nucleases within an intact cell membrane. Two apoptotic pathways have been identified by which cells can initiate and execute the cell death process: an intrinsic (mitochondria-dependent) pathway and an extrinsic (death receptor-dependent) pathway [6-8]. Intrinsic apoptosis involves the activation and mitochondrial translocation of pro-apoptotic Bcl-2 family members (*e.g*., Bax), leading to mitochondrial dysfunction and release of pro-apoptotic mediators (*e.g*., cytochrome-c).

Extrinsic apoptosis initiates with the plasma membrane assimilation of the death-inducing signaling complex (DISC), consisting of Fas, FADD, and caspase-8, by ligand-dependent (*ie*., Fas ligand, FasL) or independent mechanisms. Death receptors, a subset of type I transmembrane receptors of the tumor necrosis factor receptor family/nerve growth factor receptor family directly transduce apoptotic signals. Among these, Fas (Apo-1/CD95), is a transmembrane cell surface receptor containing three cysteine-rich extracellular domains at the amino-terminus, which are responsible for ligand binding, and an intracytoplasmic death domain (DD) of ~80 amino acids essential for transducing the apoptotic signal [9]. Binding of FasL to Fas causes a higher-order aggregation of the receptor molecules and recruitment of the adaptor molecule Fas-associated death domain (FADD) via DD-DD interactions. FADD also contains a death effector domain, which recruits pro-caspase-8 (FLICE) and/or pro-caspase-10 to the receptor. The resulting multimeric protein complex forms within seconds of receptor engagement [10]. Autoproteolytic activation of caspase-8 results in the processing of Bid to tBid, which assimilates into the mitochondria to trigger cytochrome *c *release, and may facilitate Bax activation [11].

RETRACTED

FLIP, also known as Fas-associated death domain (FADD) interleukin-1β-converting enzyme (FLICE)-like inhibitory protein has been characterized as an inhibitor of apoptosis induced by death receptors such as Fas. Multiple splice variants of c-FLIP have been found. Of these, three could be detected at the protein level. These are designated as c-FLIP short (c-FLIP_S_), c-FLIP long (c-FLIP_L_), and c-FLIP Raji (c-FLIP_R_) [12-16]. While all these isoforms of FLIP interfere with caspase-8 cleavage, only FLIP_L _is cleaved at the DISC, whereas FLIP_S _and FLIP_R _inhibit caspase-8 by remaining in the DISC. Increased levels of FLIP_L _can confer protection against Fas-induced apoptosis [12-16].

We previously reported that the expression of FLIP protected against cell death in pulmonary epithelial and endothelial cells subjected to hyperoxia [17,18], or in endothelial cells subjected to hypoxia/reoxygenation [19].

Carbon monoxide (CO) occurs in nature as a product of the combustion of organic materials. CO also arises endogenously in cells and tissues as a product of heme oxygenase (HO) activity, which degrades heme to biliverdin-IXα and ferrous iron [20]. HO-1, the inducible form of HO, responds to transcriptional upregulation by multiple forms of cellular stress. HO-1 confers cytoprotection against oxidative stress *in vitro *and *in vivo *[21]. HO-derived CO acts as a vasorelaxant and inhibits other vascular functions such as platelet aggregation and smooth muscle proliferation [22]. When applied at low concentration, CO exerts potent cytoprotective effects mimicking those of HO-1 induction, which include anti-inflammatory effects in macrophages [23,24], as well as antiapoptotic effects in vascular cells [25,26]. HO-1 and/or CO provide tissue protection in a number of *in vivo *models, including vascular injury, ischemia/reperfusion (I/R) injury, oxidative lung injury [27-32], and organ transplantation [33]. The mechanisms of CO action potentially involve modulation of intracellular signaling pathways, including activation of p38 MAPK, and soluble guanylyl cyclase [23,34,35].

Exposure to low concentrations of CO prevents the initiation of apoptosis in various cultured cells [25,36,37]. Using mouse lung endothelial cells (MLEC), we have previously demonstrated that CO treatment inhibited apoptosis in a model of hyperoxia-induced oxidative stress [37]. In the current study, we demonstrate that CO prevented Fas-activating antibody (Jo2)-induced apoptosis in MLEC by inhibition of both extrinsic and intrinsic apoptotic pathways.

## Methods

### Chemical and Reagents

Antibodies: anti-Bax, anti-caspase-8, anti-caspase-9, anti-caspase-3, anti-Fas, anti-FLIP, and protein A-agarose were from Santa Cruz Biotechnology, Inc. (Santa Cruz, CA, USA). Anti-NF-κB p65, anti-P44/42, anti-JNK and anti-FADD were from Cell Signaling Technology, Inc. (Beverly, MA). Anti-Bax 6A7 antibody was purchased from BD PharMingen (San Diego, CA). The lactate dehydrogenase (LDH) assay kit was from Roche Diagnostics Corporation (Indianapolis, IN). JNK inhibitor-II and PD 98059 were from Calbiochem (San Diego, CA). Digitonin and all other reagent chemicals were from Sigma (St. Louis, USA).

RETRACTED

### Isolation and Culture of Murine Lung Endothelial Cells

Endothelial cells were isolated by an immunobead protocol as previously described [38]. Briefly, mouse lungs were digested in collagenase and filtered through 100-μm cell strainers, centrifuged, and washed twice with medium. Cell suspensions were incubated with a monoclonal antibody (rat anti-mouse) against platelet endothelial cell adhesion molecule-1 for 30 min at 4°C. The cells were washed twice to remove unbound antibody, and resuspended in a binding buffer containing washed magnetic beads coated with sheep anti-rat immunoglobulin G. Attached cells were washed four to five times in culture medium, and then digested with trypsin/EDTA to detach the beads. Bead-free cells were centrifuged and resuspended for culture. After two passages, the cells were incubated with fluorescent-labeled diacetylated low-density lipoprotein, which is only absorbed by endothelial cells and macrophages, and sorted to homogeneity by fluorescence-activated cell sorting.

### Cell Culture and Treatments

The MLEC (passages 4-6) were cultured in Dulbecco's modified Eagle's medium (DMEM) containing 10% fetal bovine serum, 6.32 g/liter HEPES, and 3.3 ml of endothelial cell growth supplements in humidified incubators at 37°C. For Fas-activating antibody treatment, cultures were changed to serum-free medium, to which 200 ng/ml of anti-Fas antibody (Jo2) was added for the time indicated. PD 98059 from DMSO stock solution was applied at a final concentration of 25 μM for 30 min prior to Jo2 antibody treatment.

### Carbon Monoxide Exposure

Cell cultures were treated *in vitro *with CO (250 ppm) in compressed air containing 5% CO_2_, in a modular exposure chamber as previously described [23]. A CO analyzer (Interscan Corp., Chatsworth, CA) was used to measure CO levels in the chamber. For all experiments involving exposure to CO, cells were pretreated with CO for 2 h.

### Lactate Dehydrogenase (LDH) Release Assay

LDH release was measured using a commercially available assay (Cytotoxicity Detection Kit; Roche Molecular Biochemicals). After gentle agitation, 200 μl of medium was removed at various times to be used for the assay. The samples were incubated (30 min) with buffer containing NAD^+^, lactate, and tetrazolium. LDH converts lactate to pyruvate generating NADH. The NADH then reduces tetrazolium (yellow) to formazan (red), which was detected by absorbance at 490 nm.

RETRACTED

### Immunoprecipitation and Western Blot Analysis

Proteins were isolated from MLEC cultures in immunoprecipitation buffer (1 × PBS, 1% (vol/vol) Nonidet P-40, 0.5% (weight/vol) sodium deoxycholate, 0.1% (weight/vol) sodium dodecyl sulphate, 0.1 mg/ml phenylmethylsulfonyl fluoride, 30 μl/ml aprotinin, and 1 mM sodium orthovanadate). For immunoprecipitation, 1 μg of antibody (anti-Fas, anti-6A7) was added to 500 μg of total protein in 500 μl, rotated for 2 h at 4 °C, and then incubated with 20 μl of beads (protein A-sucrose, Santa Cruz Biotechnology, Inc., Santa Cruz, CA) for 2 h, spun down at 500 × g, and washed three times with immunoprecipitation buffer. Then, 20 μl of loading buffer (100 mM Tris-HCl, 200 mM dithiothreitol, 4% SDS, 0.2% bromphenol blue, and 20% glycerol) was added. For SDS-PAGE, samples containing equal amounts of protein were boiled in the loading buffer and separated on SDS-PAGE, followed by transfer to polyvinylidene difluoride membranes. The membranes were blocked with 5% nonfat milk and stained with the primary antibodies for 2 h at the optimal concentrations. After five washes in phosphate-buffered saline with 0.2% Tween 20, the horseradish peroxidase-conjugated secondary antibody was applied, and the blot was developed with enhanced chemiluminescence reagents (Amersham Biosciences, Piscataway, NJ).

### Statistical Analysis

All values are expressed as means +/- SE. Statistical significance was determined by student T-test and a value of *P *< 0.05 was considered significant.

## Results

### CO inhibits Fas activating antibody-induced apoptosis and caspase-9, -3 cleavage

The Fas-signaling pathway initiates upon stimulation with a specific ligand (Fas ligand) or an activating anti-Fas antibody, resulting in the activation of downstream caspases. We investigated the effect of CO on cell death induced by Fas-activating antibody (Jo2) in MLEC, using lactate dehydrogenase (LDH) release as a marker. As shown in Figure 1A, CO protected MLEC from Jo2-dependent cell death, relative to the air-exposed control. After 1 h of incubation with the activating anti-Fas antibody Jo2, caspase-9 and caspase-3 were cleaved in MLEC (Figure 1B). Carbon monoxide (CO) exposure delayed the activation (cleavage) of both caspases in response to Jo2 (Figure 1B), suggesting that CO inhibits Fas-dependent apoptosis in endothelial cells.

**Figure 1:** **CO inhibits cell death and caspase activation induced by Fas activating antibody Jo2**. MLEC cultures were pretreated in the absence or presence of CO (250 ppm) for 2 h prior to the addition of antibody Jo2 (200 ng/ml) for the indicated times. 200 μl of supernatant medium was removed for LDH assays as described in Methods (A). The data represent an average of two independent experiments with each sample in triplicate (n = 3). Data from Jo2 treated cells in the presence of CO were compared with control (Jo2 treatment alone) cells at each time point using Student's T-test (*P < 0.05). The total lysates were subjected to Western blot to detect caspase-9 and caspase-3. β-actin served as the standard (B). Westerns are representative of three independent experiments.

RETRACTED

### CO provides protection against extrinsic apoptosis

To investigate the mechanisms involved in the CO-dependent inhibition of Jo2-induced apoptosis, we tested the hypothesis that CO inhibits activation of extrinsic apoptotic signaling pathways. The treatment of MLEC with Jo2 induced DISC formation (Figure 2A) and activated caspase-8 (Figure 2B). When MLEC were treated with Jo2 in the presence of CO (250 ppm), the CO treatment inhibited Jo2-dependent DISC formation (Figure 2A) and caspase-8 activation (Figure 2B), relative to air-treated controls.

**Figure 2:** **CO inhibited Jo2-dependent caspase-8 and Bax activation**. MLEC cultures were pretreated in the absence or presence of CO (250 ppm) for 2 h prior to the addition of antibody Jo2 (200 ng/ml) for the indicated times. The total lysates were subjected to immunopreciptiation (IP) with anti-Fas, followed by immunoblotting (IB) to detect caspase-8. Total Fas served as the standard. The control lane (c) represents cell lysate taken immediately after Jo2 addtion (A). Lysates were subjected to Western blot analysis to detect caspase-8 (B). MLEC cultures were pretreated in the absence or presence of CO (250 ppm) for 2 h prior to the addition of antibody Jo2 (200 ng/ml) for the indicated times. Lysates were subjected to immunoprecipitation with antibody 6A7 that specifically recognizes the activated form of Bax, followed by immunoblotting with anti-Bax. Total Bax served as the standard (C). Westerns are representative of three independent experiments.

### CO inhibits Bax activation

We next tested whether an intrinsic apoptosis pathway involving Bax may participate in apoptogenic signaling pathways activated by Jo2. The treatment of MLEC with Jo2 resulted in the activation of Bax (Figure 2C), as determined by immunoprecipitation with the anti-Bax monoclonal antibody 6A7, which specifically recognizes a conformational change in Bax protein associated with its activation [38]. Bax activation is a hallmark of the intrinsic apoptosis pathway, but may also be activated secondary to extrinsic apoptosis through the caspase-8 dependent activation of Bid [17]. CO decreased Jo2-inducible Bax activation (Figure 2C) relative to air-treated controls.

RETRACTED

### CO upregulates FLIP expression and increases FLIP in the DISC

We hypothesized that CO may protect MLEC from Jo2-dependent apoptosis by regulating the expression of FLIP. In MLEC stimulated with Jo2, CO treatment upregulated FLIP_L _(Figure 3A), and increased the amount of FLIP protein associated with the DISC relative to air-treated controls (Figure 3B). These results suggest that CO, by upregulating FLIP_L _and its association with the DISC, inhibits the recruitment and activation of caspase-8.

**Figure 3:** **CO upregulated FLIP and increased DISC associated FLIP**. MLEC cultures were pretreated in the absence or presence of CO (250 ppm) for 2 h prior to the addition of antibody Jo2 (200 ng/ml) for the indicated times. The total lysates were subjected to Western blot analysis to detect FLIP (A), or to immunoprecipitation (IP) with anti-Fas followed by immunoblotting (IB) to detect FLIP. β-Actin (A) or Total Fas (B) served as the standard. Westerns are representative of three independent experiments.

### CO decreases FADD phosphorylation and its recruitment in the DISC via inhibition of JNK signaling

Treatment of MLEC with Jo2 increased the time-dependent phosphorylation of FADD (Figure 4A). Furthermore Jo2 treatment time-dependently increased the phosphorylation of FADD in association with the DISC in MLEC (Figure 4B), indicating that FADD phosphorylation may be necessary for DISC formation in MLEC. CO (250 ppm) decreased the phosphorylation of FADD in response to Jo2 stimulation, relative to air-treated controls (Figure 4A). CO also dramatically decreased FADD phosphorylation in the DISC (Figure 4B).

**Figure 4:** **CO inhibited FADD phosphorylation via blockage of JNK signaling**. MLEC cultures were pretreated in the absence or presence of CO (250 ppm) for 2 h prior to the addition of antibody Jo2 (200 ng/ml) for the indicated times. The total lysates were subjected to Western blot analysis to detect phosphorylated and total FADD (A), or to immunoprecipitation (IP) with anti-Fas followed by immunoblotting to detect phospho-FADD (B). Lysates were subjected to immunoblotting to detect phospho- and total JNK. (C). MLEC cultures were treated with antibody Jo2 (200 ng/ml) for the indicated times, in the absence or presence of JNK inhibitor (20 μM). The total lysates were subjected to immunoprecipitation with anti-Fas followed by immunoblotting to detect phospho-FADD (D). Total FADD (A, B, D) or total JNK (C) served as the standards. Westerns are representative of three independent experiments.

RETRACTED

In the presence of Jo2, CO exposure (250 ppm) time-dependently downregulated the phosphorylation of c-Jun-NH_2_-terminal kinase (JNK) in MLEC, relative to that of air-treated controls (Figure 4C). Treatment with JNK inhibitor-II (JNKi-II), an inhibitor of JNK-1/2 decreased FADD phosphorylation in the DISC (Figure 4D). The data suggest that CO inhibits FADD phosphorylation, possibly via inhibition of JNK; and that JNK-1/2 may be necessary for the phosphorylation of FADD and/or its recruitment into the DISC induced by Jo2 antibody.

### CO activates ERK1/2 and NFκB signaling

Next we tested the effect of CO on NF-κB and ERK1/2 activation in Jo2 treated MLEC. Jo2 treatment of MLEC stimulated the time-dependent phosphorylation of ERK1/2, with an apparent maximum at 12 hrs post treatment (Figure 5). Exposure to CO (250 ppm) further increased ERK1/2 activation with similar kinetics. Jo2 treatment alone did not appreciably induce NF-κB p65 phosphorylation in cells pretreated with air. On the other hand, 2 hours pretreatment with CO (250 ppm) caused a dramatic upregulation of NF-κB p65 phosphorylation at the time of Jo2 addition (0 hr), which persisted for 12 hrs **(**Figure 5**)**.

**Figure 5:** **CO activated ERK and NF-κB signaling**. MLEC cultures were pretreated in the absence or presence of CO (250 ppm) for 2 h prior to the addition of antibody Jo2 (200 ng/ml) for the indicated times. The total lysates were subjected to Western blot to detect ERK or NF-κB p65 phosphorylation. Total p65 served as the standard. Westerns are representative of three independent experiments.

We next tested the role of the ERK1/2 MAPK pathway in Jo2-mediated cell killing and in the cytoprotection afforded by CO. MLEC were treated with the ERK1/2 pathway inhibitor PD 98059, which specifically targets MEK1, the upstream regulator of ERK1/2. Treatment with PD 98059 sensitized MLEC to Jo2 mediated cell killing, and partially compromised the ability of CO to confer protection against Jo2 toxicity, as determined by LDH release assays (Figure 6A). The requirement for ERK1/2 pathway in CO-dependent suppression of apoptosis was demonstrated by Western blot analysis of caspase-3 activation. The caspase-3 cleavage induced by Jo2 in MLEC was reduced to control values by co-treatment with CO, whereas inclusion of PD 98059 abolished this effect (Figure 6B). These experiments imply a cytoprotective role for the ERK1/2 pathway against activation of the extrinsic apoptotic pathway, which is required for CO-dependent therapeutic effects (Figure 7).

RETRACTED

**Figure 6:** **CO-dependent cytoprotection requires ERK1/2 pathway**. MLEC cultures were pretreated with room air (RA) or CO (250 ppm) for 2 h prior to the addition of antibody Jo2 (200 ng/ml). Additionally, PD 98059 (25 μM) or vehicle (DMSO) was added to the cultures for 30 min prior to Jo2 addition. Cells were then incubated an additional 24 hours in the absence or presence of CO. 200 μl of supernatant medium was removed for LDH assays as described in Methods (A). The data represent triplicate (n = 3) determinations. Comparisons between the treatment groups were performed using Student's T-test (*P < 0.05). The total lysates were subjected to Western blot to detect caspase-3. β-actin served as the standard (B).

**Figure 7:** **Proposed pathways of the antiapoptotic effects of CO in Jo2-dependent apoptosis**.

## Discussion

The antiapoptotic potential of CO was first demonstrated in cell culture studies using fibroblasts or endothelial cells. Both the exogenous administration of CO or the over-expression of HO-1, inhibited TNFα-induced apoptosis in murine fibroblasts [36]. In the endothelial cell model, the inhibitory effect of CO on TNFα-induced apoptosis could be abolished with the selective chemical inhibitor, SB203580, or a p38 MAPK dominant negative mutant, implying a critical role for the p38 MAPK pathway [25]. Furthermore, HO-1 or CO co-operated with NF-κB-dependent anti-apoptotic genes (c-IAP2 and A1) to protect against TNFα-mediated endothelial cell apoptosis [39]. Exogenous CO inhibited anoxia/reoxygenation-induced apoptosis in pulmonary artery endothelial cells. This effect was associated with the activation of MKK3 and p38α MAPK, and with inhibition of Fas and FasL expression [27,30]. We have recently demonstrated that CO inhibited hyperoxia-induced endothelial cell apoptosis by downregulating ROS production, and DISC formation in MLEC [37]. In Jurkatt T cells induced to apoptosis by FasL stimulation, CO promoted, rather than inhibited FasL-dependent apoptosis, by inhibiting ERK1/2 activation [40].

The Fas-dependent apoptotic pathway has been implicated in several models of lung or vascular injury, including acute lung injury and I/R injury [41-43]. In the current study, we treated MLEC with activating anti-Fas antibody (Jo2) as a model of Fas-dependent vascular cell apoptosis. Fas is a prototype death receptor characterized by the presence of an 80 amino acid death domain in its cytoplasmic tail. This domain is essential for the recruitment of a number of signaling components upon stimulation by either activating anti-Fas antibodies or cognate FasL that initiate apoptosis. The DISC consists of an adaptor protein (such as FADD) and initiator caspases (such as caspase-8) and is essential for induction of apoptosis [9,10]. A number of proteins have been reported to regulate formation or activity of the DISC [10].

RETRACTED

The adaptor protein FADD is essential for apoptosis induced by death receptors, mediating aggregation and autocatalytic activation of caspase-8. FADD has been shown to undergo phosphorylation at Ser 194 at the G2/M transition of the cell cycle [44]. When cells are arrested in the G2-M phase of the cell cycle, they may either undergo cell death by apoptosis or necrosis or overcome the G2-M block and continue in the division cycle, often toward a post-mitotic cell death [45,46]. FADD phosphorylation plays a role in the regulation of cell growth and proliferation [44,47], and also in cellular sensitivity to apoptosis induced by anticancer drugs [48]. Currently, it remains unclear whether FADD phosphorylation is necessary for the assembly and activity of the DISC [11]. Our data suggest that FADD phosphorylation and its accumulation in the DISC is necessary for Jo2-induced apoptosis in MLEC. The kinase(s) regulating FADD phosphorylation remain unidentified [47]. In human prostate cancer cell lines, c-Jun NH_2_-terminal kinase (JNK), a member of the mitogen-activated protein kinase (MAPK) family, was associated with FADD phosphorylation [48]. Our results clearly show that CO inhibited the phosphorylation of FADD and also inhibited the activation of JNK during Jo2 stimulation. We also find that CO inhibited the apparent phosphorylation of FADD in association with Fas. It remains unclear if the phosphorylation of FADD in this context was a prerequisite for DISC formation or occurred in the context of a pre-assembled DISC. Previous studies have suggested that the phosphorylation of FADD at Ser-194 is important in the regulation of the non-apoptotic roles of FADD in regulating cell proliferation and cell cycle progression [49,50]. Nevertheless, in MLEC stimulated with Jo2 we show that the JNK inhibitor JNKi-II interfered with the detection of phospho-FADD in association with Fas in the DISC. Consistent with our observations, JNK activation has been previously implicated in the stimulation of Fas-dependent apoptosis by vanadate. In this study, JNK activation was shown to be required for Fas/FADD association [51]. Holmstrom *et al*., using the MEK1 inhibitor, have shown that ERK1/2 MAPK pathways can inhibit extrinsic apoptosis at the level of caspase-8 activation but do not inhibit Fas trafficking or DISC assembly in T cells [52]. While we propose here that CO inhibited FADD phosphorylation and DISC assembly in part through downregulation of JNK, we cannot exclude the possibility that CO also downregulated other kinases involved in FADD phosphorylation. We also cannot exclude the possibility that the effects of CO specifically on JNK phosphorylation are relevant to the activation of the non-apoptotic functions of FADD, and/or other downstream cellular targets.

RETRACTED

The results of our study also suggest the CO inhibited extrinsic apoptosis at the level of caspase-8 processing through FLIP activation. FLIP, an endogenous caspase-8 inhibitor, can block Fas-mediated apoptosis through association with the DISC [53]. Increased levels of FLIP can confer protection against Fas-induced apoptosis. FLIP_L_, FLIP_S_, FLIP_R _can be recruited to the DISC but they function differently: FLIP_S/R _prevent the initial cleavage step of caspase-8 activation between the p20 and the p10 subunit of the caspase homology domain; whereas FLIP_L _inhibits the final cleavage between the pro-domain and the p20 subunit of the p43/41 intermediate [14]. Recent studies show that PKCα/β-dependent phosphorylation regulates the ubiquitination of all c-FLIP proteins, whereas selectively prolongs the stability of the short isoforms [16]. CO upregulated FLIP_L _expression and increased the association of FLIP_L _with the DISC. Currently, we do not understand how CO upregulates FLIP expression in MLEC. We report that simultaneous application of CO during Fas-stimulation promoted the upregulation of ERK1/2 and NF-κB signaling pathways in MLEC, both of which have been implicated in FLIP regulation in other cell types [54-56]. The ERK1/2 pathway was at least in part involved in CO-dependent cytoprotection against Jo2-induced toxicity. Chemical inhibition of ERK1/2 reversed the ability of CO to downregulate Jo2-induced caspase-3 activation.

No direct evidence has been found to date that Fas-activating antibody can activate the intrinsic (Bax/mitochondria) apoptotic pathway. Injection of Jo2 antibody into *survivin*^+/- ^and *survivin*^+/+ ^mice showed that *survivin*^+/- ^mice appeared normal, but liver lysates revealed a low-level activation of caspases, with accumulation of Bax, indicating a pro-apoptotic state [57]. Here, we found that Jo2 activated Bax in MLEC. It is possible that CO inhibits Bax activation through the upregulation of FLIP, which blocks the extrinsic apoptotic pathway at the level of caspase-8 activation. We have previously shown that the vector-driven overexpression of FLIP inhibited Bax activation in MLEC during hyperoxic or hypoxia/reoxygenation stress [18,19].

## Conclusions

In summary, exogenous CO, when applied at low concentration, provides protection against Fas-activating antibody (Jo2)-induced apoptosis in MLEC by inhibiting Fas/caspase-8 and subsequently, Bax signaling pathways. FADD phosphorylation is important for DISC formation induced by Jo2. CO inhibits FADD phosphorylation and association of phospho-FADD with Fas. Although CO delayed JNK activation, the relative importance of JNK in regulating the Fas-dependent pathway remains unclear. CO increases the level of FLIP protein expression as well as its assimilation in the DISC, which inhibits the cleavage of caspase-8 (Figure 7). These results, taken together indicate that CO can protect against Fas-activating antibody-induced apoptosis by inhibiting both extrinsic (Fas/caspase-8)-dependent and intrinsic (Bax)-dependent apoptotic signaling pathways. The protection afforded by CO against activation of executioner caspase-3 was dependent on ERK1/2 pathway activation. Strategies to inhibit extrinsic apoptosis may provide therapeutic options in diseases where Fas-dependent apoptosis has been implicated in pathogenesis.

RETRACTED

## List of Abbreviations

The abbreviations used are: CO: Carbon monoxide; DISC: Death-inducing signal complex; ERK1/2: Extracellular regulated kinase-1/2; FADD: Fas-associated death domain; FBS: fetal bovine serum; c-FLIP: Fas-associated death domain interleukin-1β-converting enzyme-like inhibitory protein; c-FLIP_S_: c-FLIP short form; c-FLIP_L_: c-FLIP long form; c-FLIP_R_: c-FLIP Raji; HO-1: heme oxygenase-1; IB: immunoblotting; IP: immunoprecipitation; JNK: c-jun-NH_2_-terminal kinase; JNKi-II: inhibitor of JNK1/2; Jo2: Fas-activating antibody; LDH: lactate dehydrogenase; MAPK: mitogen activated protein kinase; MLEC: mouse lung endothelial cells; PD 98059: mitogen activated protein kinase kinase (MEK)-1 inhibitor.

## Competing interests

The authors declare that they have no competing interests.

## Authors' contributions

All authors have read and approved this manuscript. XW conceived and designed the studies, and conducted experiments; YW performed immunoblot and immunoprecipitation experiments, SJL performed revision experiments, HPK analyzed the data, AMKC supervised the studies and analyzed the data, SWR analyzed the data and wrote the manuscript.

## Authors' Information

XW performed this research as a faculty member at the University of Pittsburgh, and is currently employed by the US Food and Drug Administration; SWR is currently employed by Brigham and Women's Hospital, Boston, and is an adjunct scientist of the Lovelace Respiratory Research Institute.
